# Physio-biochemical responses and expressional profiling analysis of drought tolerant genes in new promising rice genotype

This article has been retracted.

**DOI:** 10.1371/journal.pone.0266087

**Published:** 2022-03-29

**Authors:** Haytham A. Freeg, Kotb A. Attia, Stuart Casson, Sajid Fiaz, Ebrahim A. Ramadan, Antar El- Banna, Nicholas Zoulias, Ali Aboshosha, Salman Alamery

**Affiliations:** 1 Department of Molecular Biology and Biotechnology, College of Science, Sheffield University, Sheffield, TN, United Kingdom; 2 Rice Biotechnology Lab., Rice Research & Training Center (RRTC), Field Crops Research Institute, ARC, Sakhah, Egypt; 3 Department of Genetics, College of Agriculture, Kafr-El-Sheikh University, Kafr El Sheikh, Egypt; 4 Department of Biochemistry, College of Science, King Saud University, Riyadh, Saudi Arabia; 5 Department of Plant Breeding and Genetics, The University of Haripur, Haripur, Pakistan; University of Education Lahore, Pakistan, PAKISTAN

## Abstract

Rice cultivation in Egypt is limited by the scarcity of water resources. The main strategy of rice breeders to overcome this problem is to develop new high-yielding varieties that are tolerant to drought stress. In this study, an drought-tolerant (IR60080-46A) variety was crossed with commercial Egyptian varieties using the back-cross method and marker-assisted selection (MAS) approach. The advanced lines of these crosses were selected under drought stress conditions. The best-performing candidate line, RBL-112, and its parental genotypes, were evaluated under drought stress and control conditions. The RBL-112 line showed superior its root system, which in turn produced higher grain yield under drought-stress conditions than its parental and check genotypes. Furthermore, physiological and biochemical studies showed that the RBL-112 line maintained higher relative water content (RWC), maximum quantum efficiency of photosystem II (Fv/Fm) values, proline content, superoxide dismutase (SOD) activity, and lower malondialdehyde (MDA) content compared to its parents and the check. The functional expression profiles of 22 drought tolerance-related genes were studied, out of which the genes *OsAHL1*, *OsLEA3*, *OsCATA*, *OsP5CS*, *OsSNAC1*, *Os1g64660*, *OsRab21*, *OsAPX2*, *OsDREB2A*, *OsSKIPa*, and *OsLG3* were strongly induced in the newly developed RBL-112 line under drought-stress conditions. It could be concluded that the new line has a higher capacity to modulate physiological activities and expression levels of several drought-induced genes to withstand drought stress with high yielding ability. This finding suggests that the RBL-112 line presents a promising new addition to enable sustainable rice cultivation under water-limited conditions, and confirms the efficiency of the approach implemented in the current study.

## 1. Introduction

Rice is the most important crop for approximately half of the world’s population and is cultivated under different agro-systems compared to other cereals [1]. In the Middle East, Egypt is the largest rice producer, and rice is mainly produced in the lower valley of the Nile River under flood irrigation conditions [2]. In Egypt, rice was cultivated on 360.44 thousand hectares (ha) with a total production of 3.15 million tons in 2018 [3]. This growth in production was mainly because of the development and dissemination of new high-yielding cultivars; however, this progress is threatened by the limited availability of land and water, which affects the sustainability of food production in the country [3]. Furthermore, owing to climate change, the incidence of drought events is likely to increase and will have a negative effect on water resources [4]. Drought can cause a reduction in rice yield of 21–90.6%, depending on the timing and severity of the drought [4]. Therefore, the main strategy of rice breeders is to produce more rice grains with less land and less water. The response of rice plants to drought is complex, with changes at the morphological, physio-biochemical, and molecular levels, which lead plants to reduce their growth as a survival technique under water-stress conditions [5]. Once water stress occurs, plants adopt a stress-defense mechanism by activating the antioxidant system to maintain reactive oxygen species (ROS) levels and homeostasis [6,7]. The complex antioxidant system consists of non-enzymatic compounds, such as tocopherols and ascorbic acid, and enzymes, such as catalase (CAT), superoxide dismutase (SOD), ascorbate peroxidase (APX), and glutathione reductase (GR) [8]. SOD plays a vital role in plant tolerance to harsh environments [9]. Proline also plays a vital role as an antioxidative defense molecule in protecting cells against damage associated with drought stress [10]. Malondialdehyde (MDA) is an indicator of oxidative damage resulting from abiotic stress [11,12]. However, a positive relationship has been documented between MDA content and drought tolerance in many plant species [13]. Consequently, these physiological indices (proline, SOD, MDA, and CAT) can be used as rapid and accurate methods for evaluating plant tolerance to drought stress [10,14,15]. Furthermore, plant responses to drought stress at the molecular level include stimuli perception followed by signal transduction pathways to activate the expression of drought-responsive genes, resulting in metabolic changes and drought adaptation [16]. Some of these genes are responsible for the accumulation of osmolytes, such as proline, betaine, sugars, antioxidant enzymes, water channel proteins, late embryogenesis-abundant (LEA), and membrane transporters [17], as well as transcriptional factors (TFs) that are characterized as major regulators of stress responsive genes [18]. The majority of these TFs belong to large TF families, such as bZIP, NAC, MYB, MYC, WRKY, and AP2/ERF [19]. Transcriptional profiling is a powerful approach to define candidate genes involved in stress responses via differential gene expression analysis at different times after the occurrence of drought stress in drought-tolerant and drought-susceptible genotypes [10]. The characterization of the genes involved in drought tolerance is of great importance for understanding drought resistance mechanisms in crops such as rice. These candidate genes could be used to develop MAS systems for drought tolerance in molecular breeding programs [20]. The present study aimed to develop a superior drought stress-tolerant variety using marker-aided pyramiding of multiple drought genes. The Egyptian variety Giza-178 was crossed with the Philippine drought-tolerant variety IR60080-46A and following selection and backcrossing under drought conditions, the advanced line RBL-112 was selected for analysis. Using a range of physiological, metabolic, and molecular markers, RBL-112 demonstrated improved drought tolerance and yield compared with the parental lines. This offers a promising route for sustainable rice production under drought stress.

## 2. Materials and methods

### 2.1. Plant materials and field evaluation

This study was conducted using a newly developed high yielding drought tolerant line RBL-112, selected from a fifth generation of a backcross population (BC1F5) generated from the cross between the Egyptian variety Giza-178 as the recurrent parent and a Philippines drought-tolerant variety IR60080-46A (S1 Fig). This line along with its parents and the drought sensitive variety, IR64, were utilized in this study.

### 2.2. Field evaluation under drought and normal irrigated conditions

The plant materials were exposed to two field experiments at the experimental farm of Rice Research and Training Center (RRTC), Sakha, Kafrelsheikh, Egypt (30° 57’ 12" North latitude, 31° 07’ 19" East longitude), where the weather is hot and humid. The first experiment was transplanted under normal condition (N) of continuous flooding, while the other one was transplanted under water stress regime (S) with flush irrigation every 12 days. Thirty days old seedlings of each genotype were individually transplanted in the permanent field in seven rows. Each row was five meters long and contained 25 hills by adopting a space of 20 cm. Both experiments were designed in Randomized Complete Block Design (RCBD) with three replications of the same set of genotypes. The recommended cultural practices were followed under both experiments.

At maturity, ten plants from each genotype (Giza-178, IR60080-46A, IR64 and RBL-112) in each replication were randomly selected to measure the phenotypic data, which included: days to heading (day; DH), plant height (cm; PH), panicle length (cm; PL), number of tillers per plant (NTP); panicles per plant (PP), spikelet sterility percentage (%; SS), 100-grain weight (g; 100-GW) and grain yield plant ^-1^(g; GYP). Flag leaf area (cm^2^; FLA) was measured at panicle initiation stage following the manual method proposed by [21]. Chlorophyll content (SPAD) was measured using chlorophyll analytical apparatus (chlorophyll meter SPAD-502. Konica Minolta sensing Inc. Ltd., Japan). Five flag leaves were measured from the widest part of the leaf of the main culm of each genotype in each replication. Maximum root length (cm; RL) was determined as the length of the root from the base of the plant to the tip of the main axis of the primary root. Root volume (cm^3^; RV) was determined in cubic centimeters using a standard column; root volume was taken by the water displacement method. Harvest index percentage (%; HI) was calculated using the formula reported by [22].

### 2.3. Controlled condition for physiological, biochemical and gene expression profilling

The seeds of the tested genotypes; candidate line RBL112, IR60080-46A, Giza 178, and IR64 were directly planted in 13D pots (0.88 l), (East Riding Horticulture, York, UK) containing soil consisting of 70% Kettering Loam (Boughton, UK), 23% Vitax John Innes No. 3 (Leicester, UK), 5% silica sand and 2% Osmocote Extract Standard 5–6 month slow-release fertilizer (ICL, Ipswich, UK) by volume saturated with water. Plants were grown in Conviron controlled-environment growth chambers (Controlled Environments Ltd., Winnipeg, MB, Canada). The growth conditions were: 13h 30°C: 11 h 24°C light: dark cycle, PAR 1000 μmol m^-2^ s^-1^ and 60% relative humidity, with a constant supply of water to the pot base and watering from the top once a week unless otherwise stated. The plants were grown in water-flooded trays for up to 29 days, accordingly, the stress treatment was applied by draining the water and stopping watering the plant, while the control plants remained under flooded condition.

### 2.4. Physiological and biochemical assays

#### 2.4.1. Proline content

The proline concentration was measured in fresh weight (FW) of the leaves using a standard concentration curve as μmol g^-1^ FW as described by [23].

#### 2.4.2. Superoxide Dismutase (SOD) activity

Leaf samples (1 g) were used to determine the protein content according to the method described by [24]. The SOD activity was measured using the superoxide dismutase activity Assay Kit (APEXbio Company) and the protocol described by the manufacturer was followed based on a colorimetric method with detection at 450 nm using Elisa plate reader.

#### 2.4.3. Lipid peroxidation: Malondialdehyde (MDA) content

The MDA content in rice leaves as an end product of lipid peroxidation was measured using the thiobarbituric acid (TBA) test as described by [25]. The absorbance of MDA was measured by spectrophotometer at 532 and 600 nm. The value for non-specific absorption at 600 nm was subtracted. The MDA content was calculated using the extinction coefficient 155 mM^-1^ cm^-1^.

#### 2.4.4. Fv/Fm values

Fv/FM values were measured 1 hour before the onset of the photoperiod, with a FluorPen FP 100 (PSI, Drasov, Czech Republic).

#### 2.4.5. Relative Water Content (RWC)

Leaf samples were harvested and the fresh weight (FW) was recorded. Then the leaf samples were soaked in fresh deionized water for 24h, and then placed on tissue paper to remove excess water then weighed to determine the full turgid weight (TW). Next, the leaf samples were oven-dried at 70°C for 72 h. and the dry weight (DW) was measured. The RWC was calculated using the following formula given by [26]:

RWC(%)=[(FW‐DW)/(TW‐DW)]×100.

#### 2.4.6. Stomatal impressions and counting

Ten fully expanded and healthy leaves from each genotype (leaf 5) were selected for stomata count. Dental resin (Coltene, President, light body dental resin) was applied to the abaxial surface of the leaves and allowed to set. Leaf material was removed, and impressions coated with one layer of clear nail varnish. Peels of dental resin impressions in the clear tape were placed over the clear nail varnish and mounted on to slides for microscopic imaging. A Leica DM IRBE Inverted Microscope with Planachromat 20x/ 0.41/ 0.17-A lens was used to image impressions. Micro-Manager 1.4 software was used to acquire Z-stack files of 3 points on a slide (base (b), middle (m), and tip (t)). Each Z-stack file was opened through ImageJ software, and a 400μm x 400 μm region of interest chosen for counting.


$$Stomatal\;Density\;(SD)=total\;stomata/mm^{2}.$$

### 2.5. RNA extraction, cDNA synthesises, and qRT-PCR

Total RNA was extracted from the Leaves of control and drought-stressed plants using a Quick-RNA™ MiniPrep kit (#R1055a; Zymo Research, Irvine, USA) according to the manufacturer’s instructions including an on-column DNase step. Total RNA (2μg) was reverse transcribed using the High-Capacity cDNA reverse transcription kit (#4368814; Applied Biosystems, Foster City, USA). SYBR1Green JumpStart™ Taq Ready Mix (#S5193; Sigma-Aldrich, Poole, UK) was used for qRT-PCR (3.5mM MgCl2; 375nM primer, and was performed using a CFX Connect Real-Time PCR Detection System (Bio-Rad, Watford, UK) Transcript sequences of the drought-related genes investigated were obtained from the Rice Genome Annotation Project database (http://rice.uga.edu/) then used to design gene-specific primers (S1 Table). Relative expression of target genes in the different samples was calculated from UBC1 normalized target signals using the ΔΔCT method according to [27].

### 2.6. Data analysis

The statistical analysis of the field data was done in two steps; the first one involved the ordinary analysis of variance to test the significance of the differences among the studied genotypes. The second step, the combined analysis of variance across years and environments (well-watered and drought-stress) was calculated. The test suggested by [28] was used to test the homogeneity. All statistical procedures were carried out using analysis of variance by means of ‘MSTAT” computer software package, and the means were compared based on the least significant difference (LSD) test at the 5% and 1% probability level, using three repeats. The statistical analysis of lab data was done using GraphPad prism software package.

## 3. Results

### 3.1. Effect of field drought stress on the newly developed line as compared to its parents

The study manipulated four different genotypes under two different environments, where normal irrigation and water stress conditions were applied. Analysis of variance revealed that the environment’s mean squares and the genotype x environment mean squares were highly significant for all studied traits, which demonstrated that the performance of the four genotypes differed from normal to drought-stress conditions (Table 1). The genotypes x years interaction mean squares were non-significant for all the studied traits, thus indicated that these genotypes would not be affected by the years or the performance of the tested genotypes will not change from year to year.

**Table 1:** Mean squares from analysis of variance for the studied traits over drought-stress and control conditions.

Source of variance	Years (Y)	Environments (E)	E * Y	Error (a)	Genotypes (G)	G*Y	G*E	G*E*Y	Error
d.f	1	1	1	8	3	3	3	3	24
No. of tillers / plant	0.431 ns	198.413**	1.357ns	3.091	42.369**	1.427 ns	19.594**	0.989 ns	2.125
Days to heading (day)	0.590 ns	0.267 ns	0.007 ns	7.307	203.228 **	0.667 ns	44.030**	0.474 ns	5.33
Plant height (cm)	1.479 ns	1900.663**	1.220ns	17.688	3973.853**	3.161	142.935**	1.534ns	5.234
Panicle length (cm)	0.047ns	28.444**	0.024ns	0.631	18.526**	0.835ns	3.633**	0.435 ns	0.623
Chlorophyll content (SPAD)	4.069*	164.280**	0.090 ns	5.332	35.544**	0.952ns	17.951**	1.188 ns	3.931
Flag leaf area (cm^2^)	0.908ns	521.269**	0.004ns	3.542	381.258**	0.532ns	11.414**	0.499ns	3.005
Maximum Root length (cm)	0.886ns	209.08**	1.043ns	3.42	342.19**	2.77ns	5.459*	1.613ns	1.815
Root volume (cm^3^)	2.989*	1298.33**	0.918ns	5.12	856.94**	1.62ns	95.691**	5.455 ns	3.752
No. of Panicle/ Plant	0.304 ns	269.516**	1.300 ns	2.086	28.543 **	0.582 ns	71.654 **	0.856 ns	3.583
Sterility (%)	0.496 ns	447.619**	0.513ns	7.46	95.437**	0.280ns	26.526**	0.729ns	1.889
100- grain weight (g)	0.001ns	0.329**	0.003ns	0.022	1.035**	0.001ns	0.023ns	0.003 ns	0.018
Harvest index	0.478 ns	1135.2 **	0.955 ns	4.159	406.538 **	3.131 ns	38.980 ***	0.415 ns	2.952
Grain yield / Plant (g)	1.66 ns	2656.080 **	32.637 **	2.13	393.635**	2.196 ns	320.411**	3.238*	1.381

* and ** significant at 0.05 and 0.01 levels of probability. Ns: Not significant.

We further studied the growth characters of the tested genotypes under both normal irrigation and drought stress conditions. Days to heading was significantly affected by drought-stress in the four studied genotypes (Table 2). The genotypes IR64 and Giza-178 exhibited early flowering under drought-stress compared to normal conditions, while the drought-stress caused a slight flowering delay in tolerant genotypes; for newly developed line RBL112 and its tolerant parent IR60080-46A (Table 2). It is an effective strategy to develop a short duration variety as this enables the plants to escape the terminal drought and reduces the total amount of water used during the growing season [29,30]. It was found that drought stress remarkably reduced the plant height, tiller plant^-1^, flag leaf area, panicle length, and total chlorophyll content in all rice genotypes (Table 2). Interestingly, for those traits the candidate line RBL112 exhibited the least reduction percentage as well as the most desired performance as compared to other genotypes. Drought-stress negatively affected the root length and root volume, however, the studied genotypes displayed significant differences in these two traits under normal and drought-stress conditions (Table 2). The candidate line RBL-112 showed the maximum root length and volume under drought-stress, and was more similar to those of IR60080-46 which indicated that the deep-rooted-RBL-112 line and IR60080-46A were well adapted to water-stress than other ones.

**Table 2:** Mean performance of the studied genotypes for growth traits in both environments and their combined data during the two growing seasons.

Genotypes	IR64			Giza178			IR6008046A			RBL112		
	C	D	R%	C	D	R%	C	D	R%	C	D	R%
Days to heading	114.58 a	109.02b	-5.10	105.11c	103.58cd	1.46	100.90d	103.53cd	2.54	104.71c	106.70bc	1.87
Tiller/ Plant	21.44 a	14.36d	33.02	23.62a	18.35b	22.31	17.68bc	15.45cd	12.61	18.66b	16.98bc	9.00
Plant height (cm)	101.22 c	79.31f	21.64	93.33d	87.62e	6.11	135.11a	122.06b	9.66	102.82c	93.14d	9.42
Flag leaf Area	38.31b	33.74d	11.94	28.78c	20.37f	29.23	410.25a	33.52d	16.72	34.77c	28.12e	19.12
Panicle length (cm)	21.48bc	19.17d	10.76	22.56ab	19.91cd	11.77	21.73abc	21.21bc	2.39	23.63a	22.95ab	2.84
Ch. Content (SPAD)	40.68ab	33.71c	17.13	41.68ab	37.74abc	9.46	38.13abc	36.91bc	3.21	42.09a	39.43ab	6.33
Maximum Root Length (cm)	24.54d	18.71e	23.74d	28.50c	23.66d	16.98	34.65a	31.27b	9.75	33.53a	30.59b	8.77
Root volume (cm3)	56.72d	40.96 f	27.78	66.45b	51.66e	22.25	67.54b	60.81c	9.96	70.74a	66.12b	6.54

C: Control D: Drought stress R%: Reduction percentage. Means having the same letter (s) are not significantly different while Different letters significantly different from each other according to Duncan’s multiple range test. Results are means of six replicates in two years.

The significant reduction in the grain yield and its components traits in the four tested genotypes were noticed under drought-stress conditions compared with control (Table 3). However, under the drought-stress, the candidate line RBL-112 consistently showed improved performance, even when compared to its drought-resistant parent, IR60080-46A (Table 3). Drought-stress significantly increased the sterility percentage in all the studied genotypes and was most pronounced in the drought-sensitive variety IR64. The candidate line RBL-112 showed a comparable decrease in sterility to IR6008046A but this was significantly less than the 46.91% increase in sterility observed in the Giza-178 recurrent parent (Table 3). The drought-stress reduced the 100-grain weight in all genotypes since the reduction was minimal in the candidate line RBL-112 with reduction of 3.42% (Table 3). The drought-stress caused a reduction in grain yield by 65.91% in IR64, 40.67% in Giza-178, 17.98% in RBL-112, and 14.67% in IR 60080-46A (Table 3). Concurrently, the promising line RBL112 recorded the highest mean valued for the harvest index under both normal irrigated and drought-stress conditions (Table 3).

**Table 3:** Mean performance of the studied genotypes for yield and its components traits in both environments and their combined data during the two growing seasons.

Genotypes	IR64			Giza178			IR6008046A			RBL112		
	C	D	R%	C	D	R%	C	D	R%	C	D	R%
No. of Panicle / Plant	20.45 ab	9.23 d	54.87	21.36 a	15.64 c	26.79	16.21 bc	15.87 bc	2.12	17.80 abc	16.12 bc	9.41
Sterility %	9.46 cd	19.58 a	51.66	7.49 de	14.11 b	46.91	7.71 de	11.46 bc	32.75	6.90 e	9.84 cd	29.92
100- grain weight (g)	2.31	2.03	12.19	2.48	2.30	7.39	2.68	2.58	3.67	2.90	2.80	3.42
Harvest index	34.64 c	19.83 e	42.75	39.49 b	30.07 d	23.86	37.77 bc	29.52 d	21.84	44.66 a	38.23 bc	14.39
Grain yield / Plant (g)	37.44 c	12.77 g	65.91	44.53 a	27.32 f	38.65	30.41 e	26.47 f	12.96	41.04 b	33.66 d	17.98

C: Control D: Drought stress R%: Reduction percentage. Means having the same letter (s) are not significantly different while Different letters significantly different from each other according to Duncan’s multiple range test. Results are means of six replicates in two years.

### 3.2. Effect of drought stress on genotypes physiological and biochemical charachters

The Physiological and biochemical responses were evaluated Drought stress significantly increased the SOD activity in all genotypes in comparison with normal irrigated conditions (Fig 1A). The candidate line RBL-112 and the tolerant parent IR60080-46A possessed significantly higher SOD in comparison to the sensitive chick IR64 and the recurrent parent Giza-178. While MDA content was markedly increased in the leaves of all studied genotypes under drought-stress in comparison to control plants (Fig 1B). MDA content was the highest in sensitive variety IR64 in contrast to the candidate line RBL-112 and the tolerant parent (IR6008046A) that displayed the lowest MDA content. Thus, this may imply that the drought-tolerance may be partially associated with low MDA content [31–33]. At the same time, the proline content was greatly increased in the leaves of all genotypes under drought-treatment. Nevertheless, the increase was significantly higher in the newly developed line RBL-112 and the tolerant parent IR6008046A than the sensitive check variety IR64 and the Egyptian parent Giza-178 (Fig 1C), The RWC was significantly decreased under drought-stress condition in all genotypes (Fig 1D). However, the candidate line RBL-112 followed by the parent IR6008046A exhibited higher values of RWC and showed a considerable ability to maintain a high level of water in their leaf tissues.

**Fig 1:** Physiological and biochemical characters: The SOD activity (A), MDA content (B), Proline content (C) and the RWC (D) in the leaves of the Susceptible check IR64 and the two parental genotypes (IR60080 and GIZA 178) and the candidate line under control and drought stress conditions. Values represent means ± SD. The asterisks above the bars indicate statically significant differences and different letters indicate significant differences between the lines. (P <0.001).

We investigated the abaxial stomata density in the studied genotypes and found that there were no significant differences in stomatal density among all tested genotypes under drought-stress conditions (Fig 2). It was found that the plants with reduced stomatal density were more efficient to conserve more water and to survive under drought-stress [34].

**Fig 2:** Abaxial stomata density in the four genotypes under drought stress conditions. Values represent means of n = 10 ± SEM (one way ANOVA).

Fv/Fm is the maximum quantum yield for primary photochemistry (photosystem-II) and dark-adapted Fv/Fm chlorophyll fluorescence values are considered to be an index of the damage to photosystem-II caused by abiotic stresses [35]. Our study found that a gradual decline in the Fv/Fm values was observed in all studied genotypes three days after the onset of drought. However, the newly developed line RBL-112 showed a higher Fv/Fm ratio and maintained Fv/Fm levels for at least a day longer than the other genotypes, which supports our findings, that the newly developed line RBL-112 exhibit more tolerance to drought stress (Fig 3).

**Fig 3:** Dark adapted Fv /Fm values over drought period in the four genotypes. One way ANOVA were performed to compare values for each day. Asterisks indicate statically significant differences p < 0.01.

### 3.3. Expressional profiles of stress-related genes in studied rice genotypes

Drought have a complex signaling network that is interconnected to each other. Several studies have reported the key player genes in drought response in various plant species. In the current study we analyzed the response of the expression patterns of, 22 drought related genes:4 drought functional genes, 4 genes encoding antioxidant enzymes and 14 transcription factors genes (S1 Table), to drought stress as compared to normal conditions in the four tested genotypes.

#### 3.3.1. Expression profiles of drought functional genes

The expression profile of the drought functional genes *OsRab21*, *OsP5CS*, *OsLEA3* and *OsHSP101* for the tested genotypes under both conditions is presented in Fig 4. Results indicated that there was an increase in the expression level for those genes in response to drought as compared to their expression under normal condition in all studied genotypes except for the OsHSP101 in the case of the sensitive check IR64 only where expression inhibition was noticed. Furthermore, under all conditions those genes expressed in the newly developed line, RBL-112, higher than its recurrent parent Giza178. (S1 Fig). We further investigated the expression pattern of the genes *OsAPX2*, *OsCATA*, *Os04g55710*, and *Os1g64660*. It was evident from the results of our study that, the expression of those genes has upregulated significantly in both the newly developed line and its tolerant parent IR60080-46A. In contrary, the expression of the genes *Os04g55710*, and *Os1g64660* were decreased in response to drought stress in the case of the sensitive check, IR64. Interestingly, the plant ascorbate peroxidases encoding gene, *OsAPX2*, was slightly expressed under normal conditions while drought stress stimulate its expression. Moreover, the The expressional level of *Os04g55710* in response to drought treatment was inhibited in IR64 and Giza178. In contrary, it was slightly induced in IR60080-46A, and remains unchanged in the candidate line RBL112, at the same time, *Os1g64660* was upregulated in the leaves of Giza178,RBL112 and IR60080-46A.

**Fig 4:** The expression level of *OsRab21* (A), *OsP5CS* (B), *OsLEA3* and *OsHSP101* (D), under normal and drought-stress conditions. Data are represent as means ± SEM, (n = 6).

#### 3.3.2. Expression profiles of transcription factors genes

Beside the drought functional and responsive genes, there are other drought regulatory important genes which so called TF genes. These TFs were found to play a critical role on up-regulating modulating down stream drought functional or responsive genes. In this regard, several genes which categorized under the TF gene families; AREB, DREB, MYB, WRKY, NAC, and bZIP were studied. The TF genes, *OsAHL1*, *OsLG3*, *OsSKIPa*, *OsZIP23 OsWRKY13*, *OsNAC1*, *OsDREB2A* and *OsDREB1C* were strongly up regulated in response to drought treatment, especially in the leaves of the tolerant genotypes namely the candidate line RBL112 and the parent IR6460080-46A. In contrast, the expression level of the TF genes *OsCDPK7*, *OsCPK4*, *OsMYB6*, *OsDREB1A and OsDREB2B* were down regulated under drought conditions in the studied genotypes except for *OsCPK4* and *OsDREB1A* were slightly induced in the sensitive check IR64. The *OsDREB2E* was differentially expressed among the four genotypes; however, it was poorly expressed under both conditions. The expression level of *OsDREB2E* gene was induced in the sensitive check IR64, remained unchanged in Giza178 and the candidate line RBL-112 with non-significant reduction in IR6008046A

In this study, we analyzed the expressional profiles of 22 genes reported to be associated with drought-tolerance in many plant species representing in (S3 Fig). Expression profiles of drought functional genes: Drought caused high induction in the expression level of the stress-responsive gene *OsRab21* in the leaves of the tolerant parent IR6008046A and the candidate line RBL-112. While it was slightly repressed in the leaves of the parent Giza-178 with no significant change in IR64 check variety compare to normal conditions (Fig 4A). This suggested that this gene is positively correlated with stress tolerance. Similarly, the gene *OsP5CS* was highly induced in the leaves of all studied genotypes under drought stress. However, the expression level was much higher in the drought-tolerant genotypes than the sensitive check IR64 and the moderate tolerant parent Giza-178 (Fig 4B). Under drought-stress, there was a massive induction in the transcriptional level of *OsLEA3* in the leaves of all studied genotypes in comparison to control conditions. However, the expression level was significantly higher in the leaves of the candidate line RBL112 (Fig 4C). The results obtained in this study indicate the crucial role of the LEA genes in drought tolerance in rice. Inhibition of rice heat shock protein gene *OsHSP101* expression was observed in the leaves of the sensitive check IR64 under drought-stress, while it was up-regulated in the leaves of the other genotypes (Fig 4D). Additionally, the parent IR6008046A scored the highest induction level (2.61 fold changes) of gene OsHSP101 expression (Fig 4D).

Expression patterns of genes encoding antioxidant enzymes: Data revealed that the OsAPX2 was very weakly expressed in the genotypes under normal conditions, while it was strongly expressed under drought-stress. Moreover, it was higher in the leaves of the tolerant genotypes than the sensitive check IR64 under drought-stress (Fig 5A). This result suggested that the APX has a major role in rice drought tolerance. The expressional level of *OsCATA* was strongly enhanced in the leaves of all studied genotypes due to drought-treatment. However, the expression level of *OsCATA* was significantly higher in the candidate line RBL-112 (15.9 fold), IR6008046A (15.7 Fold) and Giza-178 (13.9fold) in compare to IR64 (6.6 fold) (Fig 5B). The expressional level of *Os04g55710* in response to drought treatment was down regulated in IR64 and Giza-178. On the other hand, it was slightly induced in IR60080-46A, and remains unchanged in the candidate line RBL-112 (Fig 5C). While, it was higher in the drought-tolerant parent IR6008046A than the other studied genotypes under both control and drought-stress (Fig 5C). In terms of *Os1g64660* gene was highly induced in the candidate line RBL-112, IR6008046A, and Giza-178, while it was slightly repressed in IR64 under drought-stress conditions (Fig 5D). The candidate line RBL-112 showed a high level of mRNA of Os1g64660 may be it inherited this allele from the tolerant parent.

**Fig 5:** The expression level of OsAPX2 (A), OsCATA (B), Os0g557710 and Os1g64660 (D); under normal and drought-stress conditions. Data are represent as means ± SEM, (n = 6).

Expression profiles of transcription factors genes: The expression of *OsAHL1* gene was induced in the four genotypes under drought-stress. However, it was pronounced in the candidate line RBL-112 and surpassed its two parents IR6008046A and-Giza-178 (Fig 6A). This might be attributed to additive effect of the genes inherited from the both parents. While the susceptible chick IR64 scored the lowest increase. The transcript of *OsLG3* in response to drought was up regulated in the leaves of the studied genotypes. The extent of the induction was highest in the candidate line RBL-112, followed by IR6008046A, whereas, it was slightly induced in IR64 under drought-stress in comparison with non-stress conditions (Fig 6B). The expressional level of *OsSKIPa* in response to drought-stress was not altered in the leaves of IR64 and Giza-178, while it was highly expressed in IR6008046A and the candidate line RBL-112 (Fig 6C). This suggested that *OsSKIPa* has important role in drought tolerance in rice. The expressional level of *OsCDPK7* was down regulated in all genotypes with a slight reduction in the candidate line RBL-112 in response to drought-stress (Fig 7A). This result indicates that *OsCDPK7* has not major role in drought response in the studied genotypes. Similarly, the transcription levels of *OsCPK4* (a member of calcium-dependent protein kinases) was slightly up-regulated in IR64, repressed in the tolerant parent IR6008046A, and slightly down-regulated in the candidate line RBL-112 and the Giza-178 under drought (Fig 7B). These results indicate that the *OsCPK4* gene has no role in drought tolerance in neither IR6008046A nor the candidate line RBL-112. The transcription level of OsZIP23 was the highest in sensitive chick IR64, while it was poorly expressed in the other genotypes under normal growth conditions. Meanwhile, the transcript level of OsZIP23 was up-regulated in the four studied genotypes due to drought-stress (Fig 7C). The current data in (Fig 7D) displays that *OsMYB6* gene was highly repressed in the candidate line RBL-112 and the tolerant parent IR6008046A. It was slightly down-regulated in the susceptible check IR64, but it was none significantly induced in the parent Giza-178 under drought-stress compared to control conditions. These results may clarify that the candidate line RBL-112 might inherited the allele of *MYB6* locus from the tolerant parent and this allele has no important role in drought tolerance in these genotypes. In comparison with control conditions, *OsWRKY13* was strongly induced in all studied genotypes in response to drought-stress. However, it was the highest in the candidate line RBL-112, while, it was lowest in Giza-178 (Fig 7E). The stress-responsive *OsSNAC1* (a member of NAC, T.F family) displayed a highly up-regulation in the leaves tissue of the studied genotypes under drought-stress conditions. The induction extent was significantly higher in the candidate line RBL-112, IR60080-46A and Giza-178 in compare to IR64 (Fig 7F).

**Fig 6:** The expression level of *OsAHL1* (A), *OsLG3* (B), and *OsSKIPa* (D); under normal and drought-stress conditions. Data are represent as means ± SEM, (n = 6).

**Fig 7:** The expression level of *OsCDPK7* (A), *OsCPK4* (B), *OsZIP23* (C), *OsMYB6* (D), *OsWRKY13* (E) and OsNAC1 (F) under normal and drought stress conditions. Data are represent as means ± SEM (n = 6).

Expression patterns of DREBs Genes: The expression analysis of *OsDREB2A* was induced in the leaves of all studied genotypes under drought-stress, which was the highest in the candidate line RBL-112 under both normal and drought-stress conditions (Fig 8A). The differentially expressed of *OsDREB2A* between the candidate line RBL-112 and its two parents revealed that it might be inherited different alleles of that locus from its two parents. The *OsDREB1A* was up-regulated in the leaves of IR64 under drought-stress, while it was strongly repressed in the rest of the genotypes (Fig 8B). The obtained data suggest that *OsDRERB1A* may not have a key role in drought tolerance in rice. The transcription level of *OsDREB1C* was slightly induced in IR64 and Giza-178 genotypes; moreover it was strongly induced in IR6008046A and the candidate line RBL-112 in response to drought-stress (Fig 8C). The *OsDREB2E* was differentially expressed among the four genotypes; however it was poorly expressed under both conditions (Fig 8D). The expression level of *OsDREB2E* was induced in the sensitive check IR64, remained unchanged in Giza-178 and the candidate line RBL-112 with non-significant reduction in IR6008046A. The *OsDREB2B* was down-regulated in the all genotypes studied under dehydration conditions plus it was weakly expressed in the four genotypes under non stress and stress conditions (Fig 8E).

**Fig 8:** The expression level of *OsDREB2A* (A), *OsDREB1A* (B), *OsDREB1C* (C), *OsDREB2E* (D) and *OsDREB2B* (E); under normal and drought stress conditions. Data are represent as means ± SEM, (n = 6).

## 4. Discussion

The effect of drought stress on plants involves complex interactions, leading to yield reduction resulting from molecular, biochemical, physiological, and morphological changes in the plant [36]. The intensity of this effect varies depending on the plant genotype and growth stage, stress severity, and interaction among stressors [37]. In the current study, we investigated the physiological and biochemical responses, as well as the expression profile analysis of drought-tolerant genes in a novel and promising Egyptian rice genotype. Field evaluation showed the superiority of the newly developed RBL-112 genotype over its parent. RBL-112 was characterized by a deep root system with a high root volume compared to the recurrent parent Giza-178. Phenotypic performance regarding growth characteristics was found to be better than that of the other tested genotypes. Root and growth characteristics indicate the ability of the newly developed line to withstand drought stress with superior grain yield as compared to its corresponding parents. The physiological characteristics related to plant responses to abiotic stresses can be used as selection criteria to assess plant tolerance to abiotic stresses [14]. RBL-112 showed enhanced ROS scavenging activity compared to its parents, even the drought resistant one under drought stress conditions, as RBL-112 exhibited higher SOD activity in the leaves of the treated plants as compared to its parents, while accumulating high proline and lower MDA content compared to the Egyptian recurrent parent. SOD is an important antioxidant that plays a crucial role in protecting plants against oxidative stress caused by abiotic stress. Several studies have demonstrated that drought-tolerant genotypes display higher SOD activity than drought-susceptible genotypes in many plant species [38,39]. A lower MDA content indicates less oxidative damage occurring in the genotype as a consequence of drought stress [40,41]. Plants exposed to drought stress usually accumulate higher levels of proline in their leaves. Proline plays an essential role in osmoregulation, allowing cells to maintain higher water content [42]. Our study revealed that drought stress decreased RWC values in all genotypes, while the candidate line RBL-112 was best able to retain a high level of water in its leaf tissues. This ability to maintain RWC did not appear to be correlated with stomatal density. It has been shown that reduced stomatal density can improve drought tolerance [31,34]. We examined the stomatal density of our genotypes but did not observe any significant differences. However, this does not rule out changes in stomatal dynamics, which was not examined in this study. It is possible that RBL-112 showed enhanced stomatal responses to drought, which would be an interesting avenue for further investigation. Estimation of leaf chlorophyll concentration is one of the most efficient diagnostic tools for studying drought tolerance identification [43]. However, measurements of Fv/Fm provide information on the performance of photosystem II, which is inhibited by drought and other abiotic stressors [35]. Our investigation demonstrated that while a gradual decline in the Fv/Fm values was observed in all studied genotypes after the onset of drought, the RBL-112 line maintained higher Fv/Fm levels for at least a day longer than the other genotypes. Therefore, RBL-112 was better able to maintain photosynthetic performance under drought conditions. Drought stress tolerance in plants is associated with high levels of antioxidants, and thus a relatively higher ability to scavenge ROS resulting from drought-induced oxidative stress [38].

We further analyzed the expression profiles of 22 genes reported to be associated with drought tolerance in many plant species, including transcription factor and functional genes that encode antioxidant enzymes. The Rab gene family comprises abscisic acid (ABA) and stress-responsive genes that play key roles in many developmental processes in plants under diverse abiotic stresses [44]. Our study demonstrated that the Rab21 gene was positively correlated with stress tolerance in the variety IR6008046A and the candidate line RBL-112. These results agree with those reported previously [45,46]. It is well documented that *OsP5CS* encodes Δ-pyroroline-5-carboxylate synthase enzyme, which is involved in proline bio-synthases. In our study, the expression level of *OsP5CS* was associated with proline content under drought stress. Moreover, the tolerant genotypes accumulated markedly more proline than the sensitive genotypes. These results are inconsistent with those of [47], who also reported that *OsP5CS* transcript levels and proline content were significantly higher in the drought- and salt-tolerant genotypes than in the salt-sensitive ones. Late embryogenesis abundant (LEA) proteins are highly hydrophilic glycine-rich proteins that function as molecular chaperones to prevent the formation of damaged protein aggregates [48]. The expression of LEA was enhanced by the application of abscisic acid and abiotic stresses such as drought, cold, and salinity [49]. Our data revealed that the expression level of *OsLEA3* was the highest in the leaves of the candidate line RBL-112 compared to that in the other genotypes. These findings are consistent with the data reported that LEA genes play a central role in stress tolerance in plants, and their overexpression increases drought tolerance in transgenic plants [49]. It is well documented that accumulation of heat shock proteins (HSPs) plays a key role in abiotic stress responses in plants [50]. Our findings revealed the induction of *OsHSP101* in tolerant genotypes. The induction of many heat shock protein genes has been observed in rice under diverse abiotic stresses [51]. They function as molecular chaperones that prevent protein folding. The genes encoding antioxidant enzymes in the present study, *OsAPX2* and *OsCATA*, were found to be highly induced under dehydration stress conditions, suggesting their positive role in drought tolerance in rice. Thus, the better performance of the candidate lines RBL-112 and IR6008064A under drought stress could be associated with enhanced expression levels of *OsAPX2* and *OsCATA*. Similar results were reported in previous studies [8,52].

Additionally, *Os1g64660* was induced in the tolerant genotypes, whereas it was slightly repressed in the sensitive genotype, IR64. Echoing our findings, *Os1g64660* was previously identified as a drought-induced gene that could serve as a drought-tolerance marker in rice [53]. TFs are involved in multiple biological processes in plants and play key roles in controlling the expression of many stress-responsive genes [54]. Accordingly, we assayed the expression levels of several TF genes in the tested genotypes. Functional studies have revealed that *OsAHL1* enhances root development, plays a significant role in oxidative stress response, regulates chlorophyll content, and greatly improves drought tolerance in rice [45]. The expression of *OsAHL1* was significantly higher in the candidate line RBL-112 than in the other genotypes under drought stress, which increased its drought-tolerance ability. *OsLG3* is a transcription factor of the ethylene-responsive element-binding factor (ERF) family, which positively regulates drought tolerance in rice [55]. In this study, the transcript level of *OsLG3* was the highest in the candidate line RBL-112 under drought stress. *OsSKIPa* encodes a transcription factor that regulates the transcription of several stress-related genes. Similar to our results (Fig 6C), *OsSKIPa* was found to be induced in rice plants exposed to various abiotic stresses and phytohormone treatments [56]. It was reported that rice plants with enhanced *OsZIP23* expression demonstrated higher water content capacity, reduced membrane lipid peroxidation, and higher yield under water-stress conditions [57]. However, in our study, a high expression level of *OsZIP23* was found in all genotypes, even in the sensitive check IR64. Numerous studies have indicated that many MYB family members are positive regulators of drought tolerance in plants. However, many other MYBs are still relatively poorly characterized in rice [58]. The current study demonstrated that the *OsMYB6* gene was highly repressed in the candidate line RBL-112 and the tolerant parent, but was not significantly induced in the parent Giza-178 under drought stress compared to that under control conditions. These results indicate that the candidate line RBL-112 might have inherited the allele of the *OsMYB6* locus from the tolerant parent, and that this allele has no significant role in drought tolerance in these genotypes. Other studies have reported that *OsMYB6* expression was elevated in two-week-old rice seedlings under PEG treatments and then slowly decreased 6–12 h after treatment [58]. At the same time, *OsWRKY13* was strongly expressed in the studied genotypes under drought stress, and was the highest in the candidate line RBL-112 compared with other genotypes. These results revealed that *OsWRKY13* may play a positive regulatory role in plant response to dehydration stress; even though it was up-regulated in the susceptible check IR64, it was also highly induced in the tolerant lines. These results were in agreement with the literature [59,60]. In addition, a study reported that many genes were influenced by the transcription factor *OsWRKY13* in multiple signaling pathways, including abiotic stress, and suppression of MYB genes due to *OsWRKY13* was also observed in the same study [61]. NAC TFs are found only in plants and modulate a large number of genes involved in plant responses to stress and development [62]. Overexpression of *SNAC1* isolated from rice enhanced drought and salt tolerance in cotton and resulted in a high proline content and decreased MDA content [63]. The current investigation showed that *OsSNAC1* displayed the highest up-regulation in the candidate lines RBL-112, IR6008046A, and Giza-178 than in IR64 under drought stress. This finding supports the evidence that NACI functions as a positive regulator of drought tolerance in rice [64]. Dehydration-responsive element-binding (DREBs) are central plant TFs that modulate the expression of various stress-related genes [65]. We investigated the expression patterns of some of these rice *DREB* genes to determine which genes positively control the rice response to drought stress. *OsDREB2A* expression was induced by drought-stress, as found by [66]. In contrast, *DREB1A* and *DREB1C* are induced by cold stress [67]. However, we observed that *OsDREB1C* was weakly expressed in the control plants and was induced by drought stress. In contrast, *OsDREB2B* was reported to be induced by stress treatment [65]. However, *OsDREB2B* was found to be regulated by alternative splicing in rice [68]. Our data suggest that among the *DREB* genes in this study, *OsDREB2A* may play an important role in the response of rice to drought.

## 5. Conclusion

In our study, the candidate line RBL-112 was superior under field evaluation, had a higher yield under drought stress conditions, and maintained higher relative water content, Fv/Fm values, SOD activity, and proline content than other genotypes. Gene expression pattern analysis indicated that the candidate line RBL-112 had a higher capacity to modulate the expression levels of many drought-induced genes. This may be because of additive gene effects resulting from pyramiding of different genes and alleles inherited from both parents. The results clearly showed that *OsAHL1*, *OsLEA3*, *OsCATA*, *OsP5CS*, *OsSNAC1*, *Os1g64660OsRab21*, *OsAPX*, *OsDREB2A*, *OsSKIPa*, and *OsLG3* were strongly induced in drought-tolerant genotypes under drought-stress conditions. Furthermore, these genes could be utilized as candidate genes in MAS, allele mining, and gene pyramiding in more efficient breeding programs to develop rice cultivars that are better adapted to adverse environments. Finally, this study provides an insight into drought tolerance at the molecular level and an attempt to assess whether there is any natural genetic variation in the genes contributing to drought tolerance in rice. The RBL-112 line presents a promising new addition to enable sustainable rice cultivation under water-limited conditions and confirms the efficiency of the approach implemented in the current study.

## Supporting information

S1 Fig Diagram for description of candidate line RBL112 drived from back-cross population between Egyptian variety Giza-178 as a recurrent parent and a Philippines drought-tolerant variety IR60080-46A. (DOCX)

S2 Fig Leaf impression showing stomata distribution on abexial surface of (1) IR64, (2) Giza178, (3) IR608046A and (4) Candidate line RBL-112. (DOCX)

S3 Fig Heatmap analysis representing the expressional profiles of 22 gene response to drought in four studied genotypes under drought-stress and normal conditions. (DOCX)

S1 Table Gene- specific primers used in qRT-PCR. (DOCX)
